This article has been retracted.

# A paradigmatic approach to the topological measure of babesiosis drugs and estimating physical properties via QSPR analysis

**DOI:** 10.1016/j.heliyon.2024.e41615

**Published:** 2025-01-03

**Authors:** Nadeem Ul Hassan Awan, Muhammad Usman Ghani, Sakeena Bibi, Syed Ajaz K. Kirmani, Manal Elzain Mohamed Abdalla

**Affiliations:** a Department of Mathematics, Ghazi University, 32200, D.G. Khan, Pakistan; b Institute of Mathematics, Khwaja Freed University, Rahim Yar Khan, Pakistan; c Department of Mathematics, The University of Faisalabad, 38000, Faisalabad, Pakistan; d Department of Electrical Engineering, College of Engineering, Qassim University, Buraydah, 52571, Saudi Arabia; e College of Since and Art, Department of Mathematics, King Khalid University, Mahayil, Saudi Arabia

**Keywords:** Drugs, Chemical Structure, Linear QSPR model, Degree based topological indices

## Abstract

New developments in the field of chemical graph theory have made it easier to comprehend how chemical structures relate to the graphs that underlie them on a more profound level using the ideas of classical graph theory. Chemical graphs can be effectively probed with the help of quantitative structure-property relationship (QSPR) analysis. In order to statistically correlate physical attributes. Earlier research on medications motivated us to explore the quantitative structure-property relationships (QSPR) of babesiosis. We examined the babesiosis drugs data and used topological indices to do this. A measurement that reflects the theoretical characteristics of drugs is a topological index. The chemical structures of drugs that relieve pain are studied using well-known degree-based topological indices. Mepron, azithromycin, clindamycin, imidocarb, triclosan and other medications are among them. These drugs are administered to minimize or eliminate the discomfort that is felt in the affected location. The chemical structure of a molecule is represented as a graph. Further research into topological indices' QSPR analysis revealed so as a substantial link with the physical characteristics of drugs utilized in the production of drugs to halt the disease. The analysis of topological indices served as evidence for this. The results demonstrate how well the QSPR experiments on applying regression technique are useful in development of novel drugs for babesiosis and predict the characteristics of babesiosis drugs. The usefulness of applying TIs in this situation is demonstrated by the linear regression model's minimum error and correct prediction of these attributes.

## 1 Introduction

Babesia are parasitic protozoans which seem like malaria and reproduce inside of mammalian red blood cells. They have a complicated life cycle with numerous stages and morphological forms and they are mainly sustained in nature by trade with different mammals and Ixodes ticks. Victor Babes is identified the first Babesia species made the discovery in 1888. Since then, the genus has seen the discovery of more than 100 unique species, however only a small number of these are presently understood to be human. The occasionally dangerous zoonosis in the United States. The disease originally emerged in North America in the late 1960s on Nantucket Island. South and Eastern Asia, Europe, North and South America and Babesiosis have all been recorded. Babesia is spread by the bite of Ixodes scapularis ticks which are also the carriers of Lyme disease. Babesiosis in humans is a newly reported infectious disease and is protozoan types of the genus Babesia and shares significant clinical characteristics with malaria. In 1957, the first human instance was reported [1]. The epidemiology of human babesiosis has evolved since past 50 years in the northeastern United States. Asia, Europe, and South America all record sporadic instances. Majority of healthy persons only have a mild-to-moderate illness, the severity of infection can range from an asymptomatic infection to a fatal condition. The risk of developing a severe illness is higher in people over 50 and those who are immunocompromised, such as those who have cancer, HIV, lack a spleen or are on immunosuppressive medications [2]. Canine babesiosis is a widespread and found all over the world including India. It is frequent canine vector-borne diseases. Based on size, there are two main Babesia species [3]. A variety illness and characterized by pallor, fever, splenomegaly, jaundice, collapse and weakness linked to hypoxic injury, hemolysis, systemic inflammation, thrombocytopenia and pigmenturia [4]. A protozoan illness known as babesiosis results in a malaria-like condition when it parasitizes erythrocytes. Despite being a serious disease in cattle, it can also have serious health consequences for humans. People have contracted the illness in North America in the west coast, the upper midwest, the northeast mainland, and the islands off the country's northeast coast. Diseases like these are becoming more prevalent outside of their endemic or acquisition areas as a result of a highly mobile population. This is the first babesiosis case ever discovered in Canada, to our knowledge [5]. The patient, who required blood transfusions frequently throughout life, had been receiving pegylated interferon therapy for 40 weeks. Following a tainted blood transfusion, she was diagnosed with babesiosis, which was purportedly caused by an infection with Babesia microti (B. microti).

Clindamycin and quinine were used to treat her, but she passed away three days after being admitted. The second patient was an Indiana woman, age 73, who had previously undergone a liver transplant, a splenectomy, and blood transfusions. She was diagnosed with 6 % parasitemia after being hospitalized due to fever, black urine, and jaundice. She received more blood transfusions, clindamycin/quinine treatment, and treatment for increased parasitemia (by 50 %), but she did not improve [6]. Molecules can be mathematically modeled using chemical graph theory in order to examine their physical properties. Chemical structures should also be characterized. Since Topological indices are atomic descriptors that can be employed to depict these attributes and explicit substance graphs [7]. The topological indices of a drug are a mathematical worth or continuation of a given design viable that shows physical and chemical properties of a compound particle structure [8]. The significant objective of this study project is to look at the framework's most significant parts for the anticipation of babesiosis drugs. Without the requirement for compound trial and error, the topological record processing procedure is being used to evaluate the restorative attributes and biochemical information of novel drugs, which is especially invited in immature countries. The results use edge division techniques as a theoretical foundation for a topological index and make up for the lack of chemical and medical experiments. As of late, there diagram invariants (TIs) are used in Quantitative Design Property Connections (QSPR) studies. Drug bioactivity can be predicted using the Zagreb, Wiener, and Randic indices. The molecular structure of medications and their chemical properties like their boiling and melting points have been clearly linked in numerous studies. Gao et al. [9] center was around a group of shrewd polymers that is habitually utilized in the making of anticancer drugs. QSPR models food in choosing the best relationship among TIs and actual properties. Research-based therapeutic cures are being tried as drugs by researchers. In this paper, we determined degree-based TIs for babesiosis drugs. In a similar vein, the drugs used to treat babesiosis are organic molecules on which the specified topological indices are meticulously defined and measured using QSPR analysis. The investigation with linear regression shows this method is highly correlated with the characteristic of babiosis drugs TIs and drug properties has good relation.

## 2 Material and methods

In this analysis, the construction of a medication is addressed as a graph, where every vertex V(G) communicates a particle and each edge E(G) addresses a synthetic association between these atoms. It is assumed that all graphs are linked and simple. The quantity of edges that interface a vertex to different edges decides its degree. Refer to the following book [26] in cases where notations and terminologies are unclear. The degree of a vertex in a graph G is denoted by $d_{u}$ and it will represent number of vertices adjacent to it. The valence in chemistry and degree of a vertex in a graph are notions that are intricately related [28]. We used the following TIs: Degree-based topological indices which are the first and second Zagreb index (M1) [10], The KCD1(G) and KCD2(G) index [11], The first degree based TI is Randic index RA(G) calculated by Milan Randic in 1975 [12], Harmonic index is investigated in Ref. [13], Hyper Zagreb index [14], atom-bond connectivity index [15], inverse sum indegree index ABC [16] and Forgotten index [17] are studied. As a consequence, linear regression model is best to check and practice for the aforementioned examination. We endorse readers read the following articles [30] for more information on degree-based topological indices. Several bacterial infections can be treated with azithromycin, a macrolide antibiotic. Having a lengthy half-life and strong tissue penetration, azithromycin is a broad-spectrum macrolide antibiotic. In 1991, the FDA gave its approval. It is typically used to treat respiratory, enteric and genitourinary infections and it can sometimes be used in place of other macrolides to treat various enteric and infections. Patients with mild to moderate infections brought on by susceptible strains of the bacteria should take azithromycin, according to the recommended dosage. Clindamycin is used to treat severe infections brought on by anaerobic, streptococcaland pneumococcal bacteria.

It has been used off-label to treat toxoplasmosis and babesiosis because it seems to have some anti-protozoan activity. Also suggested for the treatment of severe infections brought on by anaerobic bacteria that are susceptible, as well as pneumococci and streptococci that are susceptible, in both oral and parenteral forms. Pneumocystis jirovecii pneumonia (PCP) prevention and treatment, as well as malaria caused by Plasmodium falciparum, are both indicated uses for the antibiotic atovaquone. Atovaquone possesses antibacterial and antipneumocystis action and is a hydroxynaphthoquinone or an analog of ubiquinone. Antimalarial procedures make use of it. Trypanocidal substance is diminazene are also useful in nature. A urea derivative called imidocarb is used in veterinary medicine as an antiprotozoal medication to treat infections with Babesia and other parasites. In a therapeutic environment, triclosan is used to halt the spread of bacteria. It is frequently used as a preservative and antibacterial agent in domestic items including plastic chopping boards, sporting goods. Quinine has been utilized as antipyretic and analgesic. It was frequently used as a flavoring and bitter agent, and it is still effective in the treatment of babesiosis. Its antimalarial effects' mechanisms are not fully known. The original tetracycline antibiotic and the one that is most frequently used in veterinary medicine is chlortetracycline. Artesunate is recommended for the initial management of severe malaria. As the first line of treatment for severe malaria, the World Health Organization suggests artesunate. The requirement for a more hydrophilic derivative of artemisinin led to the creation of artesunate. Tetracycline antibiotic oxytetracycline is used to treat a wide range of bacterial illnesses that are susceptible to it. A tetracycline analog used in a wide range of therapeutic disorders that was isolated from the actinomycete Streptomyces remous. Because it passively diffuses across porin channels in the bacterial membrane and is lipophilic, oxytetracycline can easily pass through cell membranes. Siddiqui et al. [18] mad a contribution towards titanium that mathematical modeling gives us a proficient method for changing over an issue from application region like science, physical science and science into a numerical system. Titanium exists in four kinds of oxides various applications exist in textures, papers, food varieties and medication. Titanium dioxide is a synthetically steady and climate well-disposed oxide that exists in unmistakable translucent stages like rutile, brookite, anatase, baddeleyite, columbite and fluorite. Thermodynamic properties of titanium dioxide were discovered to provide a deeper understanding of the chemical structure of titanium dioxide. The research on novel drugs in treatment of was discussed by Havare [19] and gave suggestion that drug discovery need huge cost to develop and intricate process so are efficiently predicted with this technique. QSPR modeling of blood cancer drugs was investigated by Nasir et al. [20] and observed as a suitable model for it. Being and efficient and vide spread QSPR studies for various TIs for drugs structures inspired us to work on current research problem. The objective of this study is thoroughly investigation on the implementation of TIs in determining the physical properties and its QSPR modeling of babiosis disease drug in healing management.

Diabetes disease drugs were discussed by Parveen et al. [21]. They impose degree base Tis with the aid of regression analysis and crafted well developed model for RA disease. Synthetic organizations of silicate and hexagon are very much portrayed by Kulli et al. [22] and made a near investigation of the designs. The deep behavior of the networks can be better understood with the help of these findings. A computational base method is applied Adnan et al. [23] for unequivocal degree and distance-based TIs for a few organizations. HIV is a deadly sickness all through the world since it has no legitimate fix to date whereas medications preliminaries are finished to battle the illness a proper QSPR model in carried out by Fozia et al. [24]. The QSPR demonstrating of cardiovascular medications is observed in Ref. [25] and Parveen et al. [26] achieved curvilinear QSPR learning of blood medicines and demonstrated right model for it. Zhan et al. [27] track down multiplicative Zagreb indices and found useful results of some graphs. Sobia Sultana made novel contribution in infertility treatment drugs on applying curvilinear QSPR modeling [29]. The distinctive face index proposed by Jamil et al. makes it very simple to compute the boiling point and π − electron energy of benzenoid hydrocarbons in an efficient manner [31]. The antimalarial drugs of diverse nature are investigated and significant results are mentioned by Nadeem et al. [32] that may be utilized new direction to develop novel malaria drugs in future. The work of Micheal et al. focusses on creating a QSPR model for anti-tuberculosis drugs and their many physicochemical characteristics employing distance-based topological indices [33]. Previous research on breast cancer, tuberculosis, Covid-19, skin cancer and QSPR studies of drugs inspired us to work on the current research work. The aim of study is to deeply investigate babiosis treatment drugs that pave the way to develop new drugs in therapeutic management [[34], [35], [36], [37]].

### 2.1 Degree base topological indices

**Definition. 2.1** ABC index [16] is given under:

$$ABC\left(G\right)=\sum_{uv\in E\left(G\right)}\sqrt{\frac{d_{u+}d_{v}-2}{d_{u}d_{v}}}$$

**Definition. 2.2** Randić index [12] is given under:

$$RA\left(G\right)=\sum_{uv\in E\left(G\right)}\sqrt{\frac{1}{d_{u}d_{v}}}$$

**Definition. 2.3** Zagreb indices [10] is given under:

$$M_{1}\left(G\right)=\sum_{uv\in E\left(G\right)}\left(d_{u}+d_{v}\right)\&\;M_{2}\left(G\right)=\sum_{uv\in E\left(G\right)}\left(d_{u}d_{v}\right)$$

**Definition. 2.4** Harmonic index [13] of G is given under:

$$H\left(G\right)=\sum_{uv\in E\left(G\right)}\frac{2}{d_{u}+d_{v}}$$

**Definition. 2.5** Forgotten index [17] is given under:

$$F\left(G\right)=\sum_{uv\in E\left(G\right)}\left[{\left(d_{u}\right)}^{2}+{\left(d_{v}\right)}^{2}\right]$$

**Definition. 2.6** KCD indices [11] are given under:

$$KCD1\left(G\right)=\sum_{uv\in E\left(G\right)}\left(d_{u}+d_{v}+d_{e}\right)$$

$$KCD2\left(G\right)=\sum_{uv\in E\left(G\right)}\left(d_{u}d_{v}\right).d_{e}$$

where $d_{e}=d_{u}+d_{v}-2$

**Definition. 2.6** Gourava Indices [34] is given under:

$${GO}_{1}\left(G\right)=\sum_{uv\in E\left(G\right)}\left[\left(d_{u}+d_{v}\right)+d_{u}d_{v}\right]$$

$${GO}_{2}\left(G\right)=\sum_{uv\in E\left(G\right)}\left[\left(d_{u}+d_{v}\right)d_{u}d_{v}\right]$$

Maple is utilized to calculate correct results. The calculation of other TIs listed in Table 1.

**Table 1:** The TIs values of candidate drugs.

**Name of drug**	**KCD1(G)**	**KCD2(G)**	**ABC(G)**	**RA(G)**	**M1(G)**	**M2(G)**	**GSO(G)**	**HM(G)**	**F(G)**	**GO1(G)**	**GO2(G)**
Mepron	226	430	20.62	12.56	142	172	497.70	714	370	314	892
Azithromycin	440	892	39.75	23.91	274	327	772.57	1440	786	601	1798
Clindamycin	216	412	20.24	12.70	136	161	485.97	684	362	297	844
Diminazene	160	278	15.91	10.06	102	114	222.04	482	254	216	552
Imidocarb	214	376	20.53	12.78	136	157	276.53	648	334	293	760
Triclosan	136	246	13.08	8.06	86	98	199.42	418	222	184	488
Quinine	210	400	18.96	11.71	132	161	414.18	664	342	293	832
Nerolidol	106	182	11.25	7.37	68	69	97.47	318	180	137	332
Gossypol	338	696	29.45	17.79	210	265	1059.07	1116	586	475	1470
Artesunate	248	510	21.61	12.75	154	190	348.81	818	438	344	1050
Oxytetracycline	312	682	26.15	15.20	192	248	795.61	1066	570	440	1448
Chlortetracycline	312	680	26.19	15.18	192	247	760.57	1064	570	439	1438
Amicarbalide	170	300	16.73	10.45	108	121	231.35	516	274	229	592

## 3 Main findings

### 3.1 Quantitative structure analysis and regression model

In the following section, drugs used to treat bebiosis are subjected to TIs. The connection between QSPR investigation and TIs proposes that the physicochemical attributes of the infection are profoundly associated. Thirteen meds mepron, azithromycin, clindamycin, diminazene, imidocarb, triclosan, quinine, nerolidol, gossypol, artesunate, oxytetracycline, ohlortetracycline, amicarb are utilized in the examination for bebiosis illness. The medications structures are portrayed in Fig. 1. In the study, regression analysis is used. Drug calculable design examination of eight TIs and find a best fit QSPR model for the previously mentioned drugs. Table 3 lists the nine physical properties of thirteen medicines used to treat babiosis, molar refractivity (R), polarity, complexity, molar volume (MV), enthalpy (E) and boiling point (BP). The condition of direct relapse model is as given:

(1) P=A+b(TI)

**Fig. 1:** Molecular structure of drugs.

**Table 2:** Statical parameters for ABC (G).

Property	N	A	b	r	r^2^	F	p
Boiling Point	12	121.794	20.973	.871	.758	28.171	.000
Enthalpy	12	29.335	2.978	.893	.797	35.308	.000
Flash Point	12	4.758	13.318	.837	.701	21.107	.001
Molar Refractivity	13	10.244	4.431	.962	.926	125.477	.000
Polar Surface Area	13	−11.931	5.776	.711	.505	11.214	.006
Polarity	13	3.549	1.768	.964	.929	144.593	.000
Molar Volume	12	17.158	12.950	.870	.757	31.218	.000
Molecular weight	13	25.383	17.464	.982	.963	184.503	.000
Complexity	13	−158.261	35.695	.925	.856	65.144	.000

Physicochemical property (P) of the given drug. A is constant, and b stands for regression coefficient. We implement MATLAB in order to calculate the results and equation (1) is pertinent for calculations. A linear QSPR model is used to analyze thirteen TIs of babiosis drugs and their properties. Topological indices of other drugs can be calculated by means of the identical technique as in Theorems 1 and 2 and definitions 2.1 to 2.6 and apply the technique as given in Ref. [20] and Tis of drugs is given in Table 1. Fig. 2 shows a 2D representation of calculated TIs of drugs. BY imposing equation (1), we find a diverse linear models and is elaborated below:

**Table:** 

**i. Regression models of KCD1 (G):**	**iii. Regression models of KCD2 (G):**
Boiling Point = 145.830 + 1.789 [KCD1 (G) ]	Boiling Point = 187.743 + 0.809 [KCD2 (G)]
Enthalpy = 33.555 + 0.251 [KCD1 (G)]	Enthalpy = 339.762 + 0.113 [KCD2 (G)]
Flash Point = 21.704 + 1.129 [KCD1 (G)]	Flash Point = 49.761 + 0.507 [KCD2 (G)]
Molar Refractivity = 22.361 + 0.351 [KCD1 (G)]	Molar Refractivity = 36.851 + 0.147 [KCD2 (G)]
Polar Surface Area = −1.83 + 0.482 [KCD1 (G)]	Polar Surface Area = 11.970 + 0.215 [KCD2 (G)]
Polarity = 8.514 + 0.140 [KCD1 (G)]	Polarity = 14.290 + 0.059 [KCD2 (G)]
Molar Volume = 59.100 + 0.996 [KCD1 (G)]	Molar Volume = 101.753 + 0.412 [KCD2 (G)]
Molecular weight = 58.661 + 1.439 [KCD1 (G)]	Molecular weight = 99.926 + 0.638 [KCD2 (G)]
Complexity = −99.315 + 2.994 [KCD1 (G)]	Complexity = −11.204 + 1.331 [KCD2 (G)]
**ii. Regression models of GO1 (G):**	**iv. Regression models of GO2 (G):**
Boiling Point = 149.566 + 1.282 [GO1 (G)]	Boiling Point = 194.643 + 0.386 [GO2 (G)]
Enthalpy = 34.445 + 0.179 [GO1 (G)]	Enthalpy = 41.169 + 0.053 [GO2 (G)]
Flash Point = 23.941 + 0.841 [GO1 (G)]	Flash Point = 53.684 + 0.242 [GO2 (G)]
Molar Refractivity = 25.169 + 0.245 [GO1 (G)]	Molar Refractivity = 40.561 + 0.068 [GO2 (G)]
Polar Surface Area = 0.310 + 0.343 [GO1 (G)]	Polar Surface Area = 14.906 + 0.102 [GO2 (G)]
Polarity = 9.679 + 0.098 [GO1 (G)]	Polarity = 15.788 + 0.027 [GO2 (G)]
Molar Volume = 70.433 + 0.687 [GO1 (G)]	Molar Volume = 116.125 + 0.186 [GO2 (G)]
Molecular weight = 67.198 + 1.016 [GO1 (G)]	Molecular weight = 112.461 + 0.298 [GO2 (G)]
Complexity = −85.242 + 2.126 [GO1 (G)]	Complexity = 9.942 + 0.626 [GO2 (G)]
**v. Regression models of RA (G)]**	**viii. Regression models of ABC (G)**
Boiling Point = 11.060 + 35.434 [RA (G)]	Boiling Point = 121.794 + 20.973 [ABC (G)]
Enthalpy = 27.357 + 5.065 [RA (G)]	Enthalpy = 29.335 + 2.978 [ABC (G)]
Flash Point = −4.062 + 22.650 [RA (G)]	Flash Point = 4.758 + 13.318 [ABC (G)]
Molar Refractivity = 3.352 + 7.817 [RA (G)]	Molar Refractivity = 10.244 + 4.431 [ABC (G)]
Polar Surface Area = −15.694 + 9.787 [RA (G)]	Polar Surface Area = −11.931 + 5.776 [ABC (G)]
Polarity = 0.788 + 3.118 [RA (G)]	Polarity = 3.549 + 1.768 [ABC (G)]
Molar Volume = -6.251 + 23.122 [RA (G)]	Molar Volume = 17.158 + 12.950 [ABC (G)]
Molecular weight = 7.377 + 30.104 [RA (G)]	Molecular weight = 25.383 + 17.464 [ABC (G)]
Complexity = −179.467 + 60.328 [RA (G)]	Complexity = −158.261 + 35.695 [ABC (G)]
**vi. Regression models of GSO (G)**	**ix. Regression models of HM (G)**
Boiling Point = 288.910 + 0.577 [GSO (G)]	Boiling Point = 168.712 + 0.522 [GSO (G)]
Enthalpy = 55.887 + 0.076 [GSO (G)]	Enthalpy = 36.964 + 0.073 [GSO (G)]
Flash Point = 101.616 + 0.384 [GSO (G)]	Flash Point = 37.135 + 0.328 [GSO (G)]
Molar Refractivity = 61.854 + 0.093 [GSO (G)]	Molar Refractivity = 30.693 + 0.098 [GSO (G)]
Polar Surface Area = 43.657 + 0.146 [GSO (G)]	Polar Surface Area = 5.782 + 0.140 [GSO (G)]
Polarity = 23.980 + 0.037 [GSO (G)]	Polarity = 11.845 + 0.039 [GSO (G)]
Molar Volume = 41.836 + 0.045 [GSO (G)]	Molar Volume = 83.884 + 0.415 [GSO (G)]
Molecular weight = 216.044 + 0.385 [GSO (G)]	Molecular weight = 81.940 + 0415 [GSO (G)]
Complexity = 212.199 + 0.843 [GSO (G)]	Complexity = −50.406 + 0.865 [GSO (G)]
**vii. Regression models of M1 (G)**	**x. Regression models of M2 (G)**
Boiling Point = 139.065 + 2.909 [M1 (G)]	Boiling Point = 159.849 + 2.282 [M2 (G)]
Enthalpy = 32.523 + 0.408 [M1 (G)]	Enthalpy = 36.204 + 0.316 [M2 (G)]
Flash Point = 17.084 + 1.839 [M1 (G)]	Flash Point = 30.594 + 1.440 [M2 (G)]
Molar Refractivity = 19.798 + 0.578 [M1 (G)]	Molar Refractivity = 29.536 + 0.424 [M2 (G)]
Polar Surface Area = −4.077 + 0.768 [M1 (G)]	Polar Surface Area = 4.210 + 0.605 [M2 (G)]
Polarity = 7.490 + 0.230 [M1 (G)]	Polarity = 11.444 + 0.169 [M2 (G)]
Molar Volume = 51.253 + 1.647 [M1 (G)]	Molar Volume = 85.455 + 1.172 [M2 (G)]
Molecular weight = 51.544 + 2.351 [M1 (G)]	Molecular weight = 80.501 + 1.784 [M2 (G)]
Complexity = −113.418 + 4.880 [M1 (G)]	Complexity = −60.378 + 3.751 [M2 (G)]

**Fig. 2:** 2D graph of medicines with TIs.

Table 2, Table 3, Table 4, Table 5, Table 6, Table 7, Table 8, Table 9, Table 10, Table 11, Table 12, Table 13 Represent the Statistical parameters used in QSPR models of TIs.

### 3.2 Statistical parameters and correlation determination

In this section, we track down the connection among TIs and actual properties of bebiosis illness medications, for example, prescriptions mepron, azithromycin, clindamycin, diminazene, imidocarb, triclosan, quinine, nerolidol, gossypol, artesunate, oxytetracycline, chlortetracycline, amicarbalide and this is effectively finished by forcing QSPR displaying. While TIs, b, r and N are free factor, relapse model consistent, connection coefficient and test size separately. This kind of examination can valuable to relate and choose the advancement of model. It is famous the worth of p is under 0.05 and r is more noteworthy than 0.6. As a result, it concluded that all of the properties listed in Table 2, Table 3, Table 4, Table 5, Table 6, Table 7, Table 8, Table 9, Table 10, Table 11, Table 12, Table 13 are significant. Table 1 shows their TIs processed utilizing sub-atomic design. The correlation coefficients between seven physical properties and TIs are shown in Table 3. Fig. 3 portrays the diagram among TIs and actual properties. The term “standard error estimate” refers to the measurement of variation for an observation that is calculated around the computed regression line. It analyzes the degree of precision of forecasts made about the determined relapse line in Table 13. In Table 14 connection assurance portrays the level of relationship that gives extra data about the relationship between factors. It's determined by squaring the worth of r.

**Table 3:** Correlation coefficients.

Topological Index	Correlation Coefficient								
	Boiling Point	Enthalpy	Flash Point	Refractivity	Polar surface area	Polarity	Molar Volume	Molecular weight	Complexity
ABC(G)	0.871	0.893	0.837	0.962	0.711	0.964	0.870	0.982	0.925
RA(G)	0.848	0.875	0.821	0.978	0.692	0.978	0.894	0.985	0.899
KCD1(G)	0.903	0.914	0.864	0.930	0.728	0.935	0.820	0.964	0.952
KCD2(G)	0.925	0.931	0.879	0.888	0.744	0.898	0.772	0.945	0.970
M1(G)	0.899	0.911	0.860	0.936	0.724	0.940	0.828	0.967	0.948
M2(G)	0.922	0.922	0.881	0.901	0.735	0.908	0.775	0.944	0.960
GSO(G)	0.890	0.852	0.898	0.767	0.693	0.788	0.603	0.769	0.845
HM (G)	0.917	0.925	0.874	0.907	0.739	0.915	0.793	0.954	0.965
F(G)	0.911	0.926	0.865	0.909	0.741	0.918	0.807	0.960	0.966
GO1	0.913	0.919	0.873	0.917	0.731	0.923	0.799	0.955	0.956
GO2	0.935	0.933	0.890	0.867	0.748	0.879	0.740	0.928	0.970

**Table 4:** Statically parameters for RA (G).

Property	N	A	b	r	r^2^	F	p
Boiling Point	12	111.060	35.434	.848	.719	23.025	.001
Enthalpy	12	27.357	5.065	.875	.766	29.497	.000
Flash Point	12	−4.062	22.650	.821	.674	18.604	.002
Molar Refractivity	13	3.352	7.817	.978	.956	218.933	.000
Polar Surface Area	13	−15.694	9.787	.692	.479	10.124	.009
Polarity	13	.788	3.118	.978	.956	238.912	.000
Molar Volume	12	−6.251	23.122	.894	.799	39.817	.000
Molecular weight	13	7.377	30.104	.985	.970	229.018	.000
Complexity	13	−179.467	60.328	.899	.808	46.302	.000

**Table 5:** Statically parameters KCD1 (G).

Property	N	A	b	r	r^2^	F	p
Boiling Point	12	145.830	1.789	.903	.816	39.943	.000
Enthalpy	12	33.555	.251	.914	.836	45.903	.000
Flash Point	12	21.704	1.129	.864	.746	26.414	.001
Molar Refractivity	13	22.361	.351	.930	.864	63.540	.000
Polar Surface Area	13	−1.837	.482	.728	.530	12.399	.005
Polarity	13	8.514	.140	.935	.874	76.180	.000
Molar Volume	12	59.100	.996	.820	.672	20.524	.001
Molecular Weight	13	58.661	1.439	.964	.930	92.902	.000
Complexity	13	−99.315	2.994	.952	.907	106.946	.000

**Table 6:** Statically parameters for KCD2 (G).

Property	N	A	b	r	r^2^	F	p
Boiling Point	12	187.743	.809	.925	.856	53.337	.000
Enthalpy	12	39.762	.113	.931	.866	58.208	.000
Flash Point	12	49.761	.507	.879	.772	30.477	.000
Molar Refractivity	13	36.851	.147	.888	.788	37.170	.000
Polar Surface Area	13	11.970	.215	.744	.554	13.671	.004
Polarity	13	14.290	.059	.898	.806	45.669	.000
Molar Volume	12	101.753	.412	.772	.597	14.788	.003
Molecular weight	13	99.926	.638	.945	.893	58.236	.000
Complexity	13	−11.204	1.331	.970	.941	175.582	.000

**Table 7:** Statically parameters for GO1 (G).

Property	N	A	b	r	r^2^	F	p
Boiling Point	12	149.566	1.282	.913	.834	45.074	.000
Enthalpy	12	34.445	.179	.919	.844	48.588	.000
Flash Point	12	23.941	.810	.873	.762	28.892	.000
Molar Refractivity	13	25.169	.245	.917	.842	53.109	.000
Polar Surface Area	13	.310	.343	.731	.535	12.647	.005
Polarity	13	9.679	.098	.923	.853	63.698	.000
Molar Volume	12	70.433	.687	.799	.638	17.650	.002
Molecular weight	13	67.198	1.016	.955	.912	72.398	.000
Complexity	13	−85.242	2.126	.956	.913	115.785	.000

**Table 8:** Statically parameters for GO2 (G).

Property	N	A	b	r	r^2^	F	p
Boiling Point	12	194.643	.386	.935	.875	63.075	.000
Enthalpy	12	41.169	.053	.933	.871	60.982	.000
Flash Point	12	53.684	.242	.890	.792	34.316	.000
Molar Refractivity	13	40.561	.068	.867	.753	30.406	.000
Polar Surface Area	13	14.906	.102	.748	.560	14.002	.003
Polarity	13	15.788	.027	.879	.772	37.287	.000
Molar Volume	12	116.125	.186	.740	.548	12.104	.006
Molecular weight	13	112.461	.298	.928	.862	43.639	.000
Complexity	13	9.942	.626	.970	.942	177.708	.000

**Table 9:** Statical parameters for GSO (G).

Property	N	A	b	r	r^2^	F	p
Boiling Point	12	288.910	.577	.890	.792	34.347	.000
Enthalpy	12	55.887	.076	.852	.725	23.738	.001
Flash Point	12	101.616	384	.898	.807	37.588	.000
Molar Refractivity	13	61.854	.093	.767	.589	14.322	.004
Polar Surface Area	13	43.657	.146	.693	.480	10.140	.009
Polarity	13	23.980	.037	.788	.620	17.972	.001
Surface Tension	12	41.836	.045	.603	.364	5.713	.038
Molecular weight	13	216.044	.385	.769	.591	10.009	.016
Complexity	13	212.199	.843	.845	.713	27.391	.000

**Table 10:** Statically parameters for HM (G).

Property	N	A	b	r	r^2^	F	p
Boiling Point	12	168.712	.522	.917	.842	47.873	.000
Enthalpy	12	36.964	.073	.925	.856	53.664	.000
Flash Point	12	37.135	.328	.874	.764	29.058	.000
Molar Refractivity	13	30.693	.098	.907	.822	46.190	.000
Polar Surface Area	13	5.782	.140	.739	.546	13.243	.000
Polarity	13	11.845	.039	.915	.837	56.313	.000
Molar Volume	12	83.884	.276	.793	.629	16.977	.002
Molecular weight	13	81.940	.415	.954	.910	70.987	.000
Complexity	13	−50.406	.865	.965	.930	146.735	.000

**Table 11:** Statically parameters for F (G).

Property	N	A	b	r	r^2^	F	p
Boiling Point	12	178.125	.958	.911	.831	44.200	.000
Enthalpy	12	37.885	.135	.926	.857	53.929	.000
Flash Point	12	43.850	.600	.865	.749	26.848	.001
Molar Refractivity	13	32.081	.181	.909	.826	47.570	.000
Polar Surface Area	13	7.655	.258	.741	.549	13.372	.004
Polarity	13	12.338	.072	.918	.842	58.620	.000
Molar Volume	12	83.623	.519	.807	.651	18.673	.002
Molecular weight	13	85.083	.771	.960	.922	82.980	.000
Complexity	13	−38.609	1.599	.966	.934	155.181	.000

**Table 12:** Statical parameters for M1 (G).

Property	N	A	b	r	r^2^	F	p
Boiling Point	12	139.065	2.909	.899	.808	37.774	.000
Enthalpy	12	32.523	.408	.911	.830	43.804	.000
Flash Point	12	17.084	1.839	.860	.740	25.602	.001
Molar Refractivity	13	19.798	.578	.936	.876	70.599	.000
Polar Surface Area	13	−4.077	.768	.724	.525	12.136	.005
Polarity	13	7.490	.230	.940	.884	84.093	.000
Molar Volume	12	51.253	1.647	.828	.686	21.814	.001
Molecular weight	13	51.544	2.351	.967	.935	100.924	.000
Complexity	13	−113.418	4.880	.948	.898	96.933	.000

**Table 13:** Statically parameters for M2 (G).

Property	N	A	b	r	r^2^	F	p
Boiling Point	12	159.849	2.282	.922	.850	51.008	.000
Enthalpy	12	36.204	.316	.922	.851	51.372	.000
Flash Point	12	30.594	1.440	.881	.777	31.288	.000
Molar Refractivity	13	29.536	.424	.901	.812	43.187	.000
Polar Surface Area	13	4.210	.605	.735	.540	12.926	.004
Polarity	13	11.444	.169	.908	.825	51.986	.000
Molar Volume	12	85.455	1.172	.775	.601	15.049	.003
Molecular weight	13	80.501	1.784	.944	.890	56.885	.000
Complexity	13	−60.378	3.751	.960	.921	127.680	.000

**Fig. 3:** Physicochemical properties and TIs.

**Table 14:** Standard error of estimate.

Topological Index	Standard Error of Estimate								
	Boiling Point	Enthalpy	Flash Point	Refractivity	Polar surface area	Polarity	Molar Volume	Molecular weight	Complexity
ABC(G)	100.88	12.794	74.009	10.116	44.962	3.8320	21.976	60.367	115.286
RA(G)	108.68	13.725	77.292	7.7820	46.107	3.0237	54.911	28.278	132.895
KCD1(G)	87.920	11.493	68.239	13.730	43.809	5.119	70.150	43.465	92.6300
KCD2(G)	77.904	10.388	64.632	17.144	42.665	6.349	77.844	53.787	73.6470
M1(G)	89.936	11.719	69.034	13.115	44.057	4.901	68.713	41.818	96.8310
M2(G)	79.401	10.960	63.978	16.145	43.323	6.023	77.437	54.353	85.4250
GSO(G)	93.423	14.884	59.495	23.875	46.090	8.808	18.773	105.062	162.359
HM(G)	81.561	10.758	65.825	15.707	43.050	5.826	74.619	49.194	80.0990
F(G)	84.329	107.73	67.825	15.185	42.925	5.728	72.379	45.798	78.0370
GO1	83.645	11.222	65.970	14.821	43.579	5.530	73.705	48.755	89.3430
GO2	72.450	10.180	61.701	18.523	42.381	6.879	82.436	61.050	73.2310

## 4 Conclusions

It is noted from statically boundaries applied to QSPR models and TIs that: The maximum correlated value of polarity, r = 0.979, is provided by harmonic RA (G). RA(G) file offers high corresponded benefit for molar volume r = 0.894 and for molecular weight r = 0.85. GO2(G) record offers the most extreme corresponding worth of boiling point for example r = 0.935. GO2 (G) and KCD1 (G) record portray most extreme connection coefficient of EP r = 0.933 and r = 931 respectively. Consonant KCD2(G) and GO2(G) both offers the greatest related benefit of molar refractivity r = 0.970. Table 3, Table 4, Table 5, Table 6, Table 7, Table 8, Table 9, Table 10, Table 11, Table 12, Table 13, Table 14 showcase different statical boundaries of connection be tween's seven actual properties of medication and the upsides of nine degree-based topological lists. We have carried out QSPR analysis for the physical properties of babiosis medications utilizing topological indices, such as boiling point, the extent of vaporization, complexity, etc. This is due to the widespread usage of QSPR technology to assess the properties of chemical structures. We get the conclusion that virtually all of the indices employed are useful since R is greater than 0.5 for the data set from the observation of outcomes and discussion. The highest association is observed for the attributes, and all of the aforementioned indices are judged to have equal predictive power. Overall, these indices prove to be excellent topological indices with strong predictive power for QSPR analysis of medicines for babiosis. These findings will help the pharmaceutical sector foresee the future and develop new medications.

## CRediT authorship contribution statement

**Nadeem Ul Hassan Awan:** Writing – original draft, Methodology, Data curation. **Muhammad Usman Ghani:** Supervision, Project administration, Formal analysis. **Sakeena Bibi:** Project administration, Investigation, Funding acquisition. **Syed Ajaz K. Kirmani:** Software, Conceptualization. **Manal Elzain Mohamed Abdalla:** Writing – review & editing, Investigation.

## Consent for publication

The authors authorize the publication of this manuscript.

## Data availability

All available data is presented in this article.

## Declaration of competing interest

The authors declare the following financial interests/personal relationships which may be considered as potential competing interests:Muhammad Usman Ghani reports administrative support, article publishing charges, equipment, drugs, or supplies, statistical analysis, and writing assistance were provided by Khwaja Fareed University of Engineering & Information Technology. Reports a relationship with that includes:. Has patent pending to. If there are other authors, they declare that they have no known competing financial interests or personal relationships that could have appeared to influence the work reported in this paper.
